The article "Healthcare Biclustering-Based Prediction on Gene Expression Dataset" was retracted in 2023. Reasons: signs of a paper mill; compromised peer review; unreliable results or conclusions.

# Healthcare Biclustering-Based Prediction on Gene Expression Dataset

**DOI:** 10.1155/2022/2263194

**Published:** 2022-02-22

**Authors:** M. Ramkumar, N. Basker, D. Pradeep, Ramesh Prajapati, N. Yuvaraj, R. Arshath Raja, C. Suresh, Rahul Vignesh, U. Barakkath Nisha, K. Srihari, Assefa Alene

**Affiliations:** ^1^Department of Computer Science and Engineering, HKBK College of Engineering, India; ^2^Department of Computer Science and Engineering, Sona College of Technology, India; ^3^Department of Computer Science and Engineering, M.Kumarasamy College of Engineering, Karur, India; ^4^Department of Computer Engineering, Shree Swaminarayan Institute of Technology (SSIT), India; ^5^Research and Publications, ICT Academy, IIT Madras Research Park, India; ^6^CSE, Sri Ranganathar Institute of Engineering and Technology, Coimbatore, India; ^7^CSE, Dhanalakshmi Srinivasan College of Engineering, Coimbatore, India; ^8^IT Department, Sri Krishna College of Engineering and Technology, Coimbatore, India; ^9^Department of Computer Science and Engineering, SNS College of Technology, India; ^10^Department of Chemical Engineering, College of Biological and Chemical Engineering, Addis Ababa Science and Technology University, Ethiopia

## Abstract

In this paper, we develop a healthcare biclustering model in the field of healthcare to reduce the inconveniences linked to the data clustering on gene expression. The present study uses two separate healthcare biclustering approaches to identify specific gene activity in certain environments and remove the duplication of broad gene information components. Moreover, because of its adequacy in the problem where populations of potential solutions allow exploration of a greater portion of the research area, machine learning or heuristic algorithm has become extensively used for healthcare biclustering in the field of healthcare. The study is evaluated in terms of average match score for nonoverlapping modules, overlapping modules through the influence of noise for constant bicluster and additive bicluster, and the run time. The results show that proposed FCM blustering method has higher average match score, and reduced run time proposed FCM than the existing PSO-SA and fuzzy logic healthcare biclustering methods.

## 1. Introduction

DNA microarray technologies help to measure levels of expression in experimental circumstances of thousands of genes [1]. Local patterns have motivated the large study to use pattern-based searches to deal with them. Due to its capacity to uncover hidden designs, the use of healthcare biclustering in biological data is common in the field of healthcare.

In the field analysis of gene expression data in healthcare field, in particular, healthcare biclustering is very important. Its primary objective is to be able to identify groups of genes that act equally under a subset of samples (conditions). But the pioneering literature algorithms have shown certain limitations on the quality of biclusters that were unveiled [2].

A network of biological entities, e.g., genes, proteins, and metabolists, is linked together [3]. One of the key issues in healthcare bioinformatics is analyzing and extracting biologically significant information from these entities.

The mechanism for generating a protein from the gene is gene expression. In two main steps, transcript and translation, this process happens, while transcription involves the production and processing of the resultant mRNA molecule by the enzyme RNA polymerase [4]. The concentration of mRNA in numeric values, namely, gene expression information, is measured using microarray DNA technologies. These technologies, known as DNA microarray technologies, enable the evaluation in various experimental conditions of expression levels of thousands of genes [5]. Indeed, for numerous biologists, these technologies have become indispensable tools. This is because genomes are used to control broad levels of gene expression in a particular organism.

DNA microarray was used in various areas of research, including gene discovery [6], the diagnosis of disease [7], and drug findings [8]. Microarrays are used to identify the functions of the genes and the mechanisms that underlie diseases.

In genetic engineering, gene expression is the most important stage of genotype phenotyping. Gene expression occurs when DNA is transcribed into RNA which is consistent with the process of gene synthesis information. These products are usually proteins, but the product is a functional RNA in nonprotein coding genes [9].

The number of genes in one cell varies between 2,000 and 60,000 for the eukaryotic cell depending on the organism. While the cell DNA sequence is equal in a certain organism, each cell exhibits only a subset of these genes at any given time, in keeping with the intricacies of gene expression regulation [10]. It is important that the genes are checked in several different conditions to draw meaningful conclusions from gene expression data. The analysis of gene expression includes a wide range of computer technologies that contribute to knowledge of gene-expression datasets.

The main contribution of the work involves the following:

- The authors investigate the proposed method using the experimental setup
- Further, the raw data after the microarray has been created from the initial setup gets completed
- The authors analyse various several preprocessing techniques of data, and the high level of data analysis is done with the help of computational techniques

## 2. Background

It is of most importance to unravel the transcriptional modules of genes which are coregulated through a series of experiments [11]. Of course, in many challenges in bioinformatics, the clustering technology was shown to be beneficial. In fact, researchers can collect data such as cancer, certain subtypes of tumors, and cancer survival rates (Wei et al., 2010). While the results were encouraging, clustering algorithms were used. There are two main disadvantages to clustering algorithms:

1. They take the entire set of samples into account. This is despite the fact that not all samples are subject to genes. They can instead only be applicable to a subset of samples, which are a key aspect of many problems in the field of biomedicine [12]. Therefore, both genes and conditions should be clustered simultaneously
2. Only in one group can each gene be clustered. However, many genes can be included in various clusters according to their effect in various biochemical processes [13].

Healthcare biclustering, which is one type of clustering, has palliated these inconveniences in this respect. Biclustering thus aims to identify maximum submatrices (along with biclusters) where a subset of genes is highly correlated with a variety of conditions [14]. However, healthcare biclustering is a highly combinatorial and NP-hard problem [15].

Healthcare biclustering use is common in the analysis of gene expression data, as can be seen in the literature. Below, we remember some basic definitions taken from the field of healthcare biclustering [16].

## 3. Proposed Model

The design of a microarray experiment is a procedure which comprises five main steps. A summary of the whole process of the proposed system has been elaborated in Figure 1. The process starts with a biological question that needed to be answered and ends up with the biological interpretation of the results.

1. Experimental design. This phase consists of the definition of the objectives, selecting the genes and experimental conditions under study, as well as choosing the platform, the marking methodology, and the number of replicates. In Figure 1, this phase is depicted by experimental box
2. Data generation. Raw data after the microarray has been created is obtained in this phase. This phase corresponds to data generation in Figure 1
3. Data Preprocessing. Raw data from the former step need to be preprocessed before being used. This step comprises background correction of the image, value extraction, data normalization, and data summarization. After that, the process continues with the first step if the data quality is not good enough
4. High-level analysis. After the obtainment of matrix expression, one or more statistical and computational methodologies must be performed for the purpose of collecting useful and relevant data. Although many techniques of data mining are now used on microarrays, a lot of work still remains to be done in this field

Two separate healthcare biclustering approaches are used in this analysis to identify specific gene activity in certain environments and remove the duplication of broad gene information components. Moreover, because of its adequacy, machine learning have become extensively used for healthcare biclustering. Furthermore, none of the solutions currently in place allow the user to pick the query priorities and their importance. Here, we have also worked towards developing a customizable approach to healthcare biclustering, where the user can weigh different targets according to the desired results preferences. Such goals include size, gene variation, or bicluster overlap. In fact, integrating new goals into search would also be extremely simple for the user.

Firstly, gene expression data biclusters tend to contain identical data under multiple gene expression conditions. The first thing is to identify the set of submatrices using the large average submatrix. This is based on a simple sense ranking that transcends a series width and average value. At this point, there are serious problems when information is enhanced by using the healthcare biclustering algorithm. Therefore, to increase healthcare biclustering, we use the large average submatrix. This compresses or removes irrelevant or less-correlated clustering results. The study uses FCM also to ensure that the number of rows and columns can be added to the submatrix for further calculation. The system is calculated for the accuracy of the components and the strength of the submatrices.

Secondly, a healthcare biclustering of the elements that are missing from gene expression data is done with a genetic-based simulated annealing algorithm. This approach uses a method of healthcare biclustering which is considered necessary to distinguish the information on gene expression.

### 3.1. Preliminaries

An **M** cell data matrix displays a microarray dataset by representing the level of gene expression of each cell in the matrix. With such aim, the proposed method uses a new strategy to eliminate low correlated biclusters and accepts only high-quality biclusters with larger correlation between them. In this method, the consistency of matrix element is measured using mean square residue, and further, it helps in finding the threshold value, in place of substituting the submatrix element values during the input matrix generation for subsequent clustering. The prediction of threshold value is usually processed using greedy strategy. Further, fuzzy-based ruleset helps in determining increment or decrement of the row/column in a submatrix.

### 3.2. Mean-Squared Residues

In this section, the consistency of matrix element is measured using mean-squared residue. The average values in rows and columns are expressed as below:

(1) $$\begin{array}{c} a_{iJ}=\frac{1}{\left|J\right|}\underset{j\in J}{\sum }a_{ij},\\ a_{Ij}=\frac{1}{\left|I\right|}\underset{i\in I}{\sum }a_{ij}. \end{array}$$

Average value of a matrix of row **i** and column **j** is given below:

(2) $$\begin{array}{c} a_{IJ}=\frac{1}{\left|I\right|\left|J\right|}\underset{i\in I,j\in J}{\sum }a_{ij}=a_{Ij}=\frac{1}{\left|I\right|}\underset{i\in I}{\sum }a_{iJ}=\frac{1}{\left|J\right|}\underset{j\in J}{\sum }a_{Ij}. \end{array}$$

The square matrix element residues are given below:

(3) $$\begin{array}{c} {RS}_{ij}={\left(a_{ij}-a_{Ij}-a_{iJ}+a_{IJ}\right)}^{2}. \end{array}$$

The mean-square residues (MSR) is finally estimated over a matrix element:

(4) $$\begin{array}{c} H\left(I,J\right)=\frac{1}{\left|I\right|\left|J\right|}\underset{i\in I,j\in J}{\sum }{RS}_{ij}. \end{array}$$

The average values of residue **R** of the **i**^th^ row and **C** values of the **j**^th^ column is given below:

(5) $$\begin{array}{c} R\left(i\right)=\frac{1}{\left|J\right|}\underset{i\in I,j\in J}{\sum }{RS}_{ij},\\ C\left(i\right)=\frac{1}{\left|I\right|}\underset{i\in I,j\in J}{\sum }{RS}_{ij}, \end{array}$$

where ∣*I*∣ represents rows and ∣*J*∣ represents columns.

### 3.3. Fitness Function

The final fitness function of our algorithm is shown in Equation (6). The objective is to minimize the value of each term so that large biclusters with a low transposed virtual error (TVE) value, a high gene variance and a little overlap are found. The aim is to minimize the value of every word.

(6) $$\begin{array}{c} \Phi_{B}=\frac{{VE}^{T}\left(B\right)}{{VE}^{T}\left(M\right)}+w_{s}\text{Vol}\left(B\right)+w_{ov}\text{overlap}\left(B\right)+w_{\mathrm{var}}\frac{1}{1+\text{GeneVar}\left(B\right)}. \end{array}$$

All terms are weighted, except for TVE as the benchmark. The value of TVE was, however, divided into the TVE value of the whole microarray for the healthcare biclustering. This is because the range of TVE values in each microarray depends on the values, although the algorithm tries to minimize it, when using a different microarray.

The algorithm leads to different types of biclusters according to their sizes, overlap, or variance between genes, changing the weights associated with different goals. All weights have been laid down the same way; biclusters with lower values for the relevant characteristic are lowered by a certain weight and vice versa. For example, small biclusters result in lower *w*_*s*_ values, whereas bigger *w*_*s*_ values lead to larger biclusters.

### 3.4. FCM Healthcare Biclustering

The proposed system uses FCM to check the number of columns and rows in the submatrix for calculation. FCM is developed using cost minimization function, and it is given below:

(7) $$\begin{array}{c} J\left(\theta ,U\right)=\overset{c}{\underset{i=1}{\sum }}\overset{c}{\underset{j=1}{\sum }}u_{ij}^{q}{\left\|x_{i}-\theta_{j}\right\|}^{2}. \end{array}$$

FCM operates as an iterative process and the process is given below.

Let *u*_*ij*_ be the membership degree for an input image *x*_*j*_, and it is given in the form of a cluster *C*_*j*_, *i* = 1, 2, ⋯, *N*, and *j* = 1, 2, ⋯, *c*, and then, Euclidean distance is computed of *x*_*i*_ over *θ*_*j*_′.

(8) $$\begin{array}{c} u_{ij}=\frac{1}{\sum_{k=1}^{c}{\left(\left(d\left({\overset{⟶}{x}}_{i},{\overset{⟶}{\theta }}_{j}\right)\right)/\left(d\left({\overset{⟶}{x}}_{i},{\overset{⟶}{\theta }}_{k}\right)\right)\right)}^{\left(1/\left(q-1\right)\right)}}, \end{array}$$

where *θ*_*j*_ is a representative, i.e., updated regularly using weighted vectors.

(9) $$\begin{array}{c} \theta_{j}=\frac{\sum_{i=1}^{n}{\left(u_{ij}\right)}^{q}{\overset{⟶}{x}}_{i}}{\sum_{i=1}^{n}{\left(u_{ij}\right)}^{q}}. \end{array}$$

The FCM algorithm can be terminated in a variety of ways. If the *θ*_*j*_ value or the membership grade differs slightly between two iterations, the process can be halted. However, the number of iterations is set. FCM is sensitive with outliers, and the requirement of it is mentioned as below:

(10) $$\begin{array}{c} \overset{m}{\underset{j=1}{\sum }}u_{ij}=1. \end{array}$$

Equation (10) represents the noise, and that accounts to obtain higher degree of membership in a cluster.

## 4. Performance Evaluation

This section presents the performance evaluation of the proposed FCM healthcare biclustering with existing PSO-SA healthcare biclustering and fuzzy logic healthcare biclustering. The study is evaluated in terms of average match score for nonoverlapping modules, overlapping modules through the influence of noise for constant bicluster and additive bicluster, and the run time.

Likewise, the methods are tested in terms of Garber gene expression dataset (Table 1) with 4553 genes, 66 samples, and 4 classes. The simulation is conducted in Python3.8, where the CNN is modelled in TensorFlow2.2. The implementations were run on a computer with two 2.10 GHz 6 core Intel Xeon CPUs and 126 GB of RAM memory.

Figure 2 shows the nonoverlapping modules with increasing noise levels for constant biclusters for Garber dataset. The results from the graph shows that with increased noise levels, the average match score tends to reduce in all the methods. However, the proposed FCM healthcare biclustering attains higher rate of average match score than other methods in healthcare field.

Figure 3 shows the overlapping modules with increasing overlap degree in case of constant bicluster. The results from the graph shows that with increased overlap degree, the average match score tends to reduce in all the methods. However, the proposed FCM healthcare biclustering attains higher rate of average match score than other methods in healthcare field.

Figure 4 shows the nonoverlapping modules with increasing noise levels for additive bicluster. The results from the graph shows that with increased noise levels, the average match score tends to reduce in all the methods. However, the proposed FCM healthcare biclustering attains higher rate of average match score than other methods in healthcare field.

Figure 5 shows the overlapping modules with increasing overlap degree in case of additive bicluster. The results from the graph shows that with increased overlap degree, the average match score tends to reduce in all the methods. However, the proposed FCM healthcare biclustering attains higher rate of average match score than other methods in healthcare field.

The results of run time is shown in Table 2, where the proposed method achieves reduced run time than existing method. This shows a faster response of gene expression estimation than other methods.

## 5. Conclusion

This study uses healthcare biclustering to reduce the inconveniences linked to the information clustering phase for gene expression and applied to gene expression results in the field of healthcare. Many strategies are necessary to deal with this issue and expand the search area through heuristic clustering approach.

Results of noise level for constant bicluster and additive bicluster and the results of overlapping modules show that the proposed FCM blustering is accurate in obtaining clusters than the existing methods. Further, the result shows that the run time is less in proposed FCM blustering and is accurate in obtaining clusters than the other existing methods. In the future, the proposed modelling can improvise with the several utilizations of machine learning or deep learning methods.

## Figures and Tables

**Figure 1:** Proposed FCM architecture.

**Figure 2:** Nonoverlapping modules with increasing noise levels for constant bicluster.

**Figure 3:** Overlapping modules in case of constant bicluster with increasing overlap degree.

**Figure 4:** Nonoverlapping modules for additive bicluster with increasing noise levels.

**Figure 5:** Overlapping modules in case of additive bicluster with increasing overlap degree.

**Table 1:** Dataset.

Dataset	Garber
Objects	66
Features	2
Classes	4

**Table 2:** Run time (ms).

Number of rows	PSO-SA	Fuzzy logic	Proposed FCM
4000	9.2345295	8.5186745	6.647225
8000	9.796987	8.7027515	8.160747
12000	10.594654	9.490192	8.426636
16000	11.474133	10.1958205	9.1118115
24000	12.4661035	10.492389	9.3572475
32000	13.8160015	11.760475	11.228697

## Data Availability

The datasets used and/or analyzed during the current study are available from the corresponding author on reasonable request.

## References

[1] Lopez-Fernandez A., Rodriguez-Baena D., Gomez-Vela F., Divina F., Garcia-Torres M. (2021). A multi-GPU biclustering algorithm for binary datasets. *Journal of Parallel and Distributed Computing*.

[2] Raff E., Zak R., Lopez Munoz G. Automatic YARA rule generation using biclustering.

[3] Aubert J., Schbath S., Robin S. (2021). Model-based biclustering for overdispersed count data with application in microbial ecology. *Methods in Ecology and Evolution*.

[4] Fang K., Chen Y., Ma S., Zhang Q. (2021). Biclustering analysis of functionals via penalized fusion. *Journal of Multivariate Analysis*.

[5] Fang G., Li P. (2021). On variational inference in biclustering models. *Proceedings of Machine Learning Research*.

[6] Xie J., Ma A., Zhang Y. (2020). QUBIC2: a novel and robust biclustering algorithm for analyses and interpretation of large-scale RNA-Seq data. *Bioinformatics*.

[7] Hanafi S., Palubeckis G., Glover F. (2020). Bi-objective optimization of biclustering with binary data. *Information Sciences*.

[8] Moran G. E., Ročková V., George E. I. (2021). Spike-and-slab lasso biclustering. *The Annals of Applied Statistics*.

[9] Wu Q., Hare A., Wang S. (2021). Bats: a spectral biclustering approach to single document topic modeling and segmentation. *ACM Transactions on Intelligent Systems and Technology (TIST)*.

[10] Lazareva O., Canzar S., Yuan K. (2021). BiCoN: network-constrained biclustering of patients and omics data. *Bioinformatics*.

[11] Nicholls K., Wallace C. (2021). Comparison of sparse biclustering algorithms for gene expression datasets. *Briefings in Bioinformatics*.

[12] Neves F., Finamore A. C., Madeira S. C., Henriques R. (2021). Mining actionable patterns of road mobility from heterogeneous traffic data using biclustering. *IEEE Transactions on Intelligent Transportation Systems*.

[13] Liu Z., Xiao Y., Hongsheng Y. (2021). BDBB: a novel beta-distribution-based biclustering algorithm for revealing local co-methylation patterns in epi-transcriptome profiling data. *IEEE Journal of Biomedical and Health Informatics*.

[14] Patowary P., Sarmah R., Bhattacharyya D. K. (2020). Developing an effective biclustering technique using an enhanced proximity measure. *Network Modeling Analysis in Health Informatics and Bioinformatics*.

[15] Zhou F., He K., Li Q., Chapkin R. S., Ni Y. (2020). Bayesian biclustering for microbial metagenomic sequencing data via multinomial matrix factorization. http://arxiv.org/abs/:2005.08361.

[16] Siminski K. (2021). FuBiNFS - fuzzy biclustering neuro-fuzzy system. *Fuzzy Sets and Systems*.

